The article "Detection of Snore from OSAHS Patients Based on Deep Learning" was published in 2020. Journal: J Healthc Eng.

# Detection of Snore from OSAHS Patients Based on Deep Learning

**DOI:** 10.1155/2020/8864863

**Published:** 2020-12-12

**Authors:** Fanlin Shen, Siyi Cheng, Zhu Li, Keqiang Yue, Wenjun Li, Lili Dai

**Affiliations:** ^1^Key Laboratory of RF Circuits and Systems, Ministry of Education, Hangzhou Dianzi University, Hangzhou, Zhejiang, China; ^2^The Affiliated Hospital of Hangzhou Normal University, Hangzhou, Zhejiang, China

## Abstract

Obstructive sleep apnea-hypopnea syndrome (OSAHS) is extremely harmful to the human body and may cause neurological dysfunction and endocrine dysfunction, resulting in damage to multiple organs and multiple systems throughout the body and negatively affecting the cardiovascular, kidney, and mental systems. Clinically, doctors usually use standard PSG (Polysomnography) to assist diagnosis. PSG determines whether a person has apnea syndrome with multidimensional data such as brain waves, heart rate, and blood oxygen saturation. In this paper, we have presented a method of recognizing OSAHS, which is convenient for patients to monitor themselves in daily life to avoid delayed treatment. Firstly, we theoretically analyzed the difference between the snoring sounds of normal people and OSAHS patients in the time and frequency domains. Secondly, the snoring sounds related to apnea events and the nonapnea related snoring sounds were classified by deep learning, and then, the severity of OSAHS symptoms had been recognized. In the algorithm proposed in this paper, the snoring data features are extracted through the three feature extraction methods, which are MFCC, LPCC, and LPMFCC. Moreover, we adopted CNN and LSTM for classification. The experimental results show that the MFCC feature extraction method and the LSTM model have the highest accuracy rate which was 87% when it is adopted for binary-classification of snoring data. Moreover, the AHI value of the patient can be obtained by the algorithm system which can determine the severity degree of OSAHS.

## 1. Introduction

Obstructive apnea hypopnea syndrome (hereinafter called OSAHS) not only leads to poor sleep quality but also leads to chronic hypoxemia, hypercapnia, and even high-grade central nervous system dysfunction lesions, which brings great negative impact to people. Therefore, in order to analyze the reason and sum up the diagnosis method and response treatment policy of OSAHS, more and more researchers are devoted to the research of the disease [1–3]. In clinic practice, polysomnography (hereinafter called PSG) is used to assist doctors in diagnosing OSAHS. PSG obtains multidimensional data such as heart rate, brain waves, chest vibration, blood oxygen saturation, breathing, and snoring. AHI (Apnea Hypopnea Index) value of the patient can be obtained after these data are fused with a certain algorithm and weights by monitoring the patient's breathing throughout the night [4, 5], which means the number of apnea index per hour, hypopnea index and obstructive pause, central pause, and mixed pause. However, there are two practical problems with PSG: 1. PSG requires professional medical personnel to operate, and the users must lie in the hospital for monitoring; 2. PSG affects the quality of sleep because the user needs to plug in the corresponding equipment in many parts of the body during use. If there is a technology that does not rely on large medical equipment and is comfortable for patients in daily use, it can not only improve the experience of patients when they are monitored but also help doctors more accurately grasp the long-term clinical performance of patients.

The article "Detection of Snore from OSAHS Patients Based on Deep Learning" was published in 2020. Journal: J Healthc Eng.

In recent years, scholars have proposed a variety of OSAHS disease discrimination techniques based on various symptom characteristics. Among them, A. Garde used the visual midpoint (radius and angle) distribution characteristics of SpO_2_ signals to distinguish OSAHS symptoms [6]; Kim used the patient's breathing sound signal to develop a classification of OSAHS severity model [7]; Volak made preliminary judgments on OSAHS through image recognition of children's dental features [8]; Castillo-Escario et al. develop an algorithm for detecting silence events and classifying them into apneas and hypopneas [9]. The current medical research reports show that the clinical apnea syndrome events manifestations of an adult are as follows [10, 11]. Snoring is loud and often be interrupted by an apnea event that lasts for about 10 s; then, a faint snoring sound appears during the incident. After the incident, the patient suffered from gasping, accompanied by loud snoring. The reason for the formation of OSAHS disease is the blockage of the internal cavity of the nose of patients initiated by the patient's oral and nasal diseases such as rhinitis or pharyngitis [12]. In general, snoring is the form of expression of OSAHS. In the study of snoring, the researchers first studied the technique of extracting snoring sounds from breathing sounds. For example, the nonlinear classification algorithm to identify snoring sounds was studied by Ankishan [13]; Lim proposed a snoring recognition method based on RNN [14, 15]. The study of OSAHS recognition based on snoring has also been proposed after the effective extraction of snoring signals: After extracting the time-domain features of snoring after apnea events, Temrat et al. judged the severity degree of OSAHS through distinguishing different types of snoring by the leave-one-out cross-validation technique [16]. However, the time domain features such as zero-crossing rate (ZCR), energy entropy (EE), and integrated electromyography (IEMG) extracting snoring from background noise in this paper have two problems: (1) The similar features of some audio data are not easy to be distinguished; (2) The feature dimension is too less. Therefore, in order to extract better features, researchers also introduced neural network classification methods into snoring recognition. The advantage of detecting snoring features based on deep learning is that the neural network can automatically extract features. For example, Takahiro Emoto classified snoring data related to OSAHS (SNR) based on ANN. Unfortunately, due to the limitation of the classification effect of ANN, its accuracy result can only reach 75% [17]. Moreover, the data used in this experiment is not obtained based on the test result data output in PSG which is currently the standard diagnostic procedure for obstructive sleep apnea (hereinafter called OSA) [18] but artificially annotated data by listening to the sound. Therefore, the reliability of the experiment could not be verified by the most reliable device: PSG. In addition, B. Daurai and P. Nayak detected apnea events by using three dimensions of the chest cavity, abdomen, and respiratory airflow. The equipment used for obtaining data is inconvenient to wear and may affect the quality of sleep of users [19]. In this paper, we presented a method for automatic recognition of OSAHS based on snoring sounds classification by a neural network model. Our method only used snoring sounds for recognition. Therefore data of patients could be easily collected by recording equipment. Firstly, the snoring sounds related to apnea events and nonapnea event-related snoring sounds (see Section 2.2) are identified. Secondly, the severity of the apnea event was judged by the result of snoring sound recognition. Each snoring data is converted from the time domain to the frequency domain. The MFCC features are calculated, and then the MFCC features are used as the input of a LSTM model for binary classification. The experiments result indicates that our method could realize a recognition with high accuracy.

The article "Detection of Snore from OSAHS Patients Based on Deep Learning" was published in 2020. Journal: J Healthc Eng.

## 2. Materials and Methods

### 2.1. Flow of the Proposed Method

The algorithm flow proposed in this paper is shown in Figure 1, which is divided into two steps: feature extraction and classification. After MFCC feature extraction, snoring audio data were inputted into the CNN/LSTM neural network for binary classification, and then the algorithm outputted the recognition result.

### 2.2. Feature Extraction

Figure 2 is the data derived from PSG. The results show the multidimensional data such as pulse and oxygen saturation during patient monitoring. As shown in the figure, an obstruction pause event occurs between 23 : 01 : 10–23 : 01 : 25. The blocking pause event is obtained by multidimensional data fusion. From the dimension data of snoring, the apnea event is accompanied by a very weak snoring sound, which is marked with purple in Figure 2. The snoring that appeared after the apnea event is marked with blue. Snoring sounds that occur during apnea events and after apnea events are recorded as snoring sounds related to apnea events, which are called abnormal snoring. The remaining snoring sounds related to nonapnea events are called normal snoring sounds. In order to identify the normal snoring and abnormal snoring, we firstly extracted features of snoring signals using three different feature extraction methods which are MFCC, LPCC, and LPMFCC. The flow of feature extraction is given in Figure 3.

#### 2.2.1. MFCC

MFCC (Mel Frequency Cepstral Coefficient) is a feature inspired by the event that different human ears have different hearing sensitivity to sound waves which have different frequencies. MFCC is currently widely used in the field of audio recognition. Preemphasis, framing, and windowing pretreatment are performed in the time domain before feature extraction [20]. Preemphasis is to pass the speech signal through a high-pass filter in order to compensate for the loss of high-frequency components and improve the high-frequency components. Frame is to gather N sampling points into a set unit. The purpose is to make the parameters between one frame and another frame transition smoothly. Windowing is to multiply each frame by Hamming window, which is to reduce signal characteristics leak in the frequency domain. After pretreatment, the signal is converted to the frequency domain by Fourier transform and the power spectrum is calculated. Then, the Mel-scale triangular filter bank is used to smooth the frequency spectrum instead of avoiding the characteristic parameters that are affected by the pitch of the speech. Finally, we calculate the log energy and MFCC coefficient of each filter bank output [21]. As shown in Equation (1) and Equation (2), the log energy *s*(*m*) output by each filter bank is obtained by Equation (1), where m represents the number of filters, *k* represents the number of Fourier transform points, *n* represents the order of MFCC coefficients, *Xa*(*k*) represents the power of the speech signal spectrum obtained by performing fast Fourier transform of each frame signal and taking the modulus square; *H*(*k*) represents the frequency response of the energy spectrum obtained by the triangular filter; the MFCC coefficient *C*(*n*) is obtained based on DCT (discrete cosine transform) [21]:

(1) $$\begin{array}{c} \begin{array}{c} s\left(m\right)=\ln\left(\sum_{k=0}^{N-1}{\left|Xa\left(k\right)\right|}^{2}H\left(k\right)\right),\;\;0\leq m\leq M \end{array}, \end{array}$$

(2) $$\begin{array}{c} \begin{array}{c} C\left(n\right)=\sum_{m=0}^{N-1}s\left(m\right)\cos\left(\frac{\pi n\left(m-0.5\right)}{m}\right),\;\;n=1,2,\ldots ,L \end{array}. \end{array}$$

Each piece of snoring audio was divided into frames by 0.03 s length of frame and 0.01 s shift of frame, the extracted feature dimension of which is 298 *∗* 40.

The article "Detection of Snore from OSAHS Patients Based on Deep Learning" was published in 2020. Journal: J Healthc Eng.

#### 2.2.2. LPCC

In order to obtain the basic parameters of speech signals, LPCC has become one of the main technologies to estimate the parameters of speech signals. The algorithm of LPCC is shown in Figure 1, except for the same pretreatment as shown in Section 2.2.1, the signal undergoes the current prediction model to calculate the LPC coefficients, and then is converted into LPCC coefficients in the form of the spectrum by cepstrum, *V*(*z*) is the channel transfer function. *G* is the gain of the filter, *a*_*k*_ is the set of known linear regression coefficients (LPC) autoregressive coefficients, and *p* is the order of the all-pole filter. The LPC coefficients obtained by the autocorrelation method ensure the stability of the system so that the channel model transferred function corresponding to the following Equation (3) has a minimum phase [22]. Equation (4) can deduce the recursive relationship between the cepstral *c*(*n*) of the speech signal and the LPC coefficient, where *c*(1) is the DC component and reflects the spectral energy, and its value does not affect the spectral shape. The second formula is used when the number of LPCC coefficients is not greater than the number of LPC coefficients, and the third formula is used when the number of LPCC coefficients is greater than the number of LPC coefficients:

(3) $$\begin{array}{c} , \end{array}$$

(4) $$\begin{array}{c} \left\{\begin{array}{c} c\left(n\right)=a_{n}+\overset{n-1}{\underset{k=1}{\sum }}\left(1-\frac{k}{n}\right)a_{k}c\left(n-k\right),\;\;\;1<n<p\\ c\left(n\right)=\overset{p}{\underset{k=1}{\sum }}\left(1-\frac{k}{n}\right)a_{k}c\left(n-k\right),\;\;n>p \end{array}\right. \end{array}$$

#### 2.2.3. LPMFCC

The LPMFCC feature parameters are based on LPC. The process obtained by calculating the Mel Cepstrum of LPC is shown in formula (5). Firstly, the LPC coefficients are subjected to Fourier transform, and then the LPC coefficients are obtained through DFT Discrete spectrum*X*_*a*_(*k*). Secondly, the square of the spectrum amplitude is calculated to obtain the discrete energy spectrum *X*_*a*_(*k*)^2^. Among them, N represents the number of Fourier transform points. Thirdly, a set of Mel-scale triangular filters are used to filter the discrete energy spectrum, and then the output results are subjected to logarithm operation to obtain the log energy *Z*_*a*_(*m*), as shown in Equation (6), where *H*_*m*_(*k*) (0 ≤ m ≤ *M*) is several band-pass filters, and *M* is the number of filters. Finally, the above logarithmic energy is calculated by discrete cosine transform, and a new characteristic parameter LPMFCC is obtained:

(5) $$\begin{array}{c} , \end{array}$$

(6) $$\begin{array}{c} Z_{a}\left(m\right)=\ln\left(\sum_{k=0}^{N-1}{\left|X_{a}\left(k\right)\right|}^{2}H_{m}\left(k\right)\right), \end{array}$$

(7) $$\begin{array}{c} C_{a}\left(n\right)=\sum_{m=0}^{M-1}Z_{a}\left(m\right)\cos\left[\frac{pn\left(m+\left(1/2\right)\right)}{M}\right],\;\;0\leq m\leq M. \end{array}$$

The article "Detection of Snore from OSAHS Patients Based on Deep Learning" was published in 2020. Journal: J Healthc Eng.

### 2.3. Model Recognition

#### 2.3.1. CNN-Based Audio Recognition

Research on convolutional neural networks originated in the late 19th century. Since 2012, due to breakthroughs in hardware and algorithms, both image recognition and audio recognition have made leaps and bounds [23–25]. In the field of audio recognition, Google proposed the CNN model in 2017 to identify keywords [26]. The general convolutional neural network structure usually includes a convolutional layer, a fully connected layer, and a pooling layer. The CNN model used in this article consists of a three-layer CNN structure, and the extraction result of each CNN convolutional layer is activated and connected to the Relu activation function. The max-pooling layer is finally connected to the fully connected layer to map the distributed features to the sample label space (see Figure 4), and the model parameter settings are shown in Table 1. Considering that the input MFCC features are much less complex than the image data features in image recognition, it is not necessary to adopt very deep neural networks for recognition. If the structure of the recognition model is too deep, it will result in problems such as overfitting and excessive calculation. We will conduct a comparative experiment with 3-layer CNN and 5-layer CNN to verify this viewpoint in Section 3.4, and the construction of 3-layer CNN and 5-layer CNN are shown in Tables 1 and 2.

#### 2.3.2. RNN-Based Audio Recognition

This paper also uses a recurrent neural network (RNN) model for comparing with CNN in classification performance. RNN is usually used to process a lot of sequence data {*x*_1_, *x*_2_, ... *x*_t_} and is widely used in natural language processing (NLP), speech recognition, translation, and so on. Unlike CNN, RNN has a memory function for time series, which can capture the connection and difference between the characteristics of this time point and the previous time point. RNN can be concluded as ordinary RNN and special RNN. Special RNN refers to replacing ordinary short-term memory network unit (LSTM) or gated cycle unit (GRU) with ordinary RNN unit. In this paper, the LSTM unit is used for sequence identification. As shown in Figure 5(a), from left to right in a LSTM unit structure are the forget gate, the input gate, and the output gate. The output gate controls the output of information and filters the information to be output.

The article "Detection of Snore from OSAHS Patients Based on Deep Learning" was published in 2020. Journal: J Healthc Eng.

The expression at time *t* is shown in formulae (8) to (13). *x*_*t*_ represents the input information, *h*_*t*−1_ and *h*_*t*_, respectively, represent the hidden coefficient output of the previous LSTM unit and the new LSTM unit. *C*_*t*−1_ and *C*_*t*_ represent the information output by the previous unit and the new information output by the unit,  *f*_*t*_ represents the information that the unit selectively forgets, which is multiplied with the weight *W*_*f*_  and adds to the coefficient *b*_*f*_. *i*_*t*_ and *C*_*t*_′ represent the memory information, and then are merged into *C*_*t*_, which represents the final output state shown in formula (11). *O*_*t*_ represents the state of the three gates. Then *h*_*t*_ is obtained by the multiplication of *O*_*t*_ and tanh(*c*_*t*_).

LSTM can make up for the shortcomings of ordinary RNN's short memory and uncontrollable storage content. The operation parameters of LSTM are less than the CNN parameters mentioned above, and the operation is faster, which helps avoid the gradient disappearance and explosion problems in typical RNN [27]. The RNN structure model is shown in Figure 5(b). According to the input audio spectrogram, the display dimension is *t∗f* = 298 *∗* 40 (where *t* represents time and *f* represents frequency). The input data *x*_t_ is input to the No.t RNN unit with the hidden unit *h*_*t*−1_ of the time frame output. Since one data input frame number is 298, the RNN model has 298 LSTM units, *x*_0_ ∼ *x*_297_ represents the input feature, and *y* represents the output result (see Figure 5(b)):

(8) $$\begin{array}{c} f_{t}=\theta \left(W_{f}\cdot \left[h_{t-1},x_{t}\right]+b_{f}\right), \end{array}$$

(9) $$\begin{array}{c} i_{t}=\theta \left(W_{i}\cdot \left[h_{t-1},x_{t}\right]+b_{i}\right), \end{array}$$

(10) $$\begin{array}{c} C_{t}^{\prime }=\tanh\left(W_{c}\cdot \left[h_{t-1},x_{t}\right]+b_{c}\right), \end{array}$$

(11) $$\begin{array}{c} C_{t}=f_{t}*C_{t-1}+i_{t}*C_{t}^{\prime }, \end{array}$$

(12) $$\begin{array}{c} O_{t}=\theta \left(W_{o}\cdot \left[h_{t-1},x_{t}\right]+b_{o}\right), \end{array}$$

(13) $$\begin{array}{c} h_{t}=O_{t}*tanh\left(c_{t}\right). \end{array}$$

The article "Detection of Snore from OSAHS Patients Based on Deep Learning" was published in 2020. Journal: J Healthc Eng.

## 3. Results and Discussion

### 3.1. Database

In our experiments, sleep sounds are collected from 32 volunteers (including 16 normal people and 16 OSAHS patients) through a microphone for a whole night (8 h) at a sampling frequency of 16 KHz. The device can be used at home. Snoring sounds were extracted from breathing sounds and background noise through the endpoint detection technology [27], each case of which lasting 3 s. The training samples consisted of randomly selected 16 volunteers' snoring sounds (5 normal people and 11 OSAHS patients). We classified snoring data from OSAHS patients' sleeping sounds in the whole night according to the time period displayed by the PSG picture into four categories for ready: (1) Snoring data before each apnea event; (2) Snoring data in each apnea event; (3) Snoring data after each apnea event; (4) The other snoring data in OSAHS patients' snoring data in a whole sleeping night.

### 3.2. Experimental Evidence of Data Selection

In order to verify that the snoring data which during the apnea events and behind of the apnea events have obvious characteristics differences from normal snoring data extracted from 5 normal people while sleeping at night [20], we implemented four sets of comparative experiments (see Table 3): (1) Snoring data before, during, and after apnea events and normal snoring data extracted from normal people's sleeping sounds while at night as two-class sample sets; (2) Snoring data during and after apnea events and normal snoring data extracted from normal people's sleeping sounds in the whole night as two-class sample sets; (3) Snoring data before apnea events and normal snoring data extracted from normal people's sleeping sounds in the whole night as two-class sample sets; (4) All of the snoring data extracted from OSAHS patients and normal snoring data extracted from normal people's sleeping sounds in the whole night as two-class sample sets. Each set of data is about 10000 cases and the number ratio of the two categories is 1 : 1.

Conclusions can be drawn from this experiment: the data characteristics of snoring data during the apnea events and behind of the apnea events have the most obvious differences from normal snoring data extracted from normal people's whole sleeping night.

### 3.3. Experiment

Based on the above experimental evidence in Section 3.2, the positive sample (normal snoring) is the data from the 5 normal people's whole night snoring, and the negative sample (abnormal snoring) is the data from the OSAHS patients' whole night snoring, which were taken from the apnea event's middle and behind (see Figure 2). The snoring data of the remaining 16 volunteers were used to test the generalization performance of the model (see Table 4).

The article "Detection of Snore from OSAHS Patients Based on Deep Learning" was published in 2020. Journal: J Healthc Eng.

### 3.4. Environment

The experiment in this article is operated in the ubuntu 5.4.0 environment, rtx2048 graphics card. The model is built using TensorFlow 2.0 framework. The RNN and CNN network parameters are shown in Section 2.3.

### 3.5. Evaluation

The experimental results are evaluated by 5 methods which are accuracy, sensitivity, specificity, precision, and F1-score. The expressions of these methods are given by formulae (14) to (18). In these formulas, TP presents the number of positive samples that were actually identified as positive samples; FN presents the number of the positive samples that were identified as the negative samples falsely; TN presents the number of negative samples that were correctly identified as the negative sample; FP presents the number of the negative samples that were identified as the positive sample falsely:

(14) $$\begin{array}{c} \text{accuracy}=\frac{TP+TN}{TP+TN+FP+FN}, \end{array}$$

(15) $$\begin{array}{c} \text{precision}=\frac{TP}{TP+FP}, \end{array}$$

(16) $$\begin{array}{c} \begin{array}{c} \text{sensitivity}=\text{recall}=\frac{TP}{TP+FN} \end{array}, \end{array}$$

(17) $$\begin{array}{c} \text{specificity}=\frac{TN}{TP+FP}, \end{array}$$

(18) $$\begin{array}{c} F1-\text{score}=\frac{2*\text{precision}*\text{recall}}{\text{precision}+\text{recall}}, \end{array}$$

### 3.6. Comparison of Three Feature Extraction Methods and Three Model Experiment Results

Table 5 shows the accuracy of the model test combined with the three feature extraction methods (MFCC, LPCC, LPMFCC) and the three models (3-layer CNN, 5-layer CNN, and LSTM). A horizontal comparison found that the classification effect of 5-layer CNN is the same as 3-layer CNN, and LSTM performs better than CNN in the connection and comparison of time series data features, and LSTM can make up for the shortcomings of ordinary RNNs with a short memory and uncontrollable storage content [27]. As shown in Table 5 and Figure 6, through longitudinal comparison, it is found that the feature extraction effect from the best to the worst are MFCC, LPMFCC, LPCC. This is because the LPCC algorithm has a linear prediction function for time series and can obtain more information from speech recognition [28], while MFCC maps the speech frequency to a nonlinear mel filter bank and converts it to the cepstrum domain [29]. The features extracted from the neighboring frames are almost independent and suitable for consonant recognition. The snoring sound produced by a person during sleep is caused by the blockage of the upper respiratory tract of the person due to some reason (rhinitis or pharyngitis or even cerebral nerves [30]), which causes the airflow to hit the soft tissue and generate large vibrations, like consonant. Therefore, the MFCC is more suitable for extracting a feature from snoring data in this paper.

The article "Detection of Snore from OSAHS Patients Based on Deep Learning" was published in 2020. Journal: J Healthc Eng.

### 3.7. Discussion of the Application

According to the snoring sounds data related to apnea events in 11 OSAHS patients and the whole night (about 8 hours) snoring sounds of 5 normal subjects as the test set, the LSTM model has a better classification effect than CNN, calculating the number of two types of snoring sounds from 16 volunteers' whole night after they were entered into the stored LSTM model for binary classification. Finally, calculating the AHI value according to the definition of AHI (number of sleep apnea per hour). As shown in formula (19), where AB represents the number of snoring sounds related to the apnea event (Abnormal snoring) recognized by the system, 2 represents 1 case of middle snoring sound and 1 case of posterior snore sound, and SH represents the length of sleep throughout the night. According to the AHI value, the severity of OSAHS patients can be obtained, which is divided into slight (5 ＜ AHI ≤ 15), moderate (15 ＜ AHI ≤ 30), and serious (AHI ＞ 30) [31]. As shown in Table 6(0 means no OSAHS, 1 means slight, 2 means moderate, and 3 means serious), 10 patients were tested, and the difference between the AHI which was calculated by test data and the AHI obtained by the patient through PSG actually is represented by squared different (SORT-AHI) shown in Table 6. It can be known from the table that the model has better recognition performance for the severity of OSAHS.

(19) $$\begin{array}{c} AHI=\frac{AB}{2}/SH. \end{array}$$

## 4. Conclusions

In this study, the detection of OSAHS was quantified and evaluated using the feature extraction method and deep learning algorithm. We compared the differences in detection accuracy between three feature extraction methods and three neural networks. It is found that the MFCC performs best in feature extraction and the LSTM performs better than the CNN in classification, and the combination of MFCC and LSTM performed the best, in which the accuracy of classification reached 0.87. In addition, the model can not only judge whether someone else has OSAHS through snoring but also can detect the severity degree by AHI coefficient (see Table 5), and the model has solved the problem that PSG has. However, the accuracy of the system in this study is not very well. We are going to improve the performance of the system by producing a better neural network model in the feature.

The article "Detection of Snore from OSAHS Patients Based on Deep Learning" was published in 2020. Journal: J Healthc Eng.

## Figures and Tables

**Figure 1:** The flow of the proposed method.

**Figure 2:** Data presented on PSG.

**Figure 3:** Three methods of feature extraction.

**Figure 4:** CNN architecture used in this paper.

**Figure 5:** RNN-based audio recognition. (a) LSTM cell structure. (b) LSTM neural network model.

**Figure 6:** Accuracy of three feature extraction methods and three models. (a) Accuracy of MFCC method. (b) Accuracy of LPMFCC method. (c) Accuracy of LPCC method.

**Table 1:** Parameters of our 3 layers CNN.

Block	Layer	Filter size	Filters (layer number)	Stride (step number)
Conv1 block	Conv1 maxPool1	20*∗*8	64	2
		2*∗*2		2

Conv2 block	Conv2 maxPool2	10*∗*4	64	2
		2*∗*2		2

Conv3 block	Conv3 maxPool3	5*∗*2	64	1
		2*∗*2		2

**Table 2:** Parameters of our 5 layers CNN.

Block	Layer	Filter size	Filters (layer number)	Stride (step number)
Conv1 block	Conv1 maxPool1	20*∗*8	64	2
		2*∗*2		2

Conv2 block	Conv2 maxPool2	10*∗*4	64	2
		2*∗*2		2

Conv3 block	Conv3 maxPool3	5*∗*2	64	1
		2*∗*2		2

Conv4 block	Conv4 maxPool4	2*∗*2	64	1
		2*∗*2		2

Conv5 block	Conv5 maxPool5	2*∗*2	64	1
		2*∗*2		2

**Table 3:** Results of four groups of experiments.

Test group (number)	Sensitivity	Specificity	Precision	Accuracy
1	0.75	0.75	0.50	0.60
2	0.83	0.84	0.82	0.82
3	0.42	0.53	0.43	0.48
4	0.40	0.50	0.40	0.45

**Table 4:** Data distribution.

Subjects	16 people		16 people
Class	Training set	Validation set	Test set
Normal snoring(case)	5156	516	2065
Abnormal snoring (case)	5156	516	2065

**Table 5:** Accuracy of three feature extraction methods and three models.

Feature extraction method	Evaluation	3 layers-CNN	5 layers-CNN	LSTM
MFCC	Sensitivity	0.83	0.82	0.84
	Specificity	0.84	0.81	0.91
	Precision	0.82	0.84	0.91
	Accuracy	0.82	0.85	0.87
	F1-score	0.82	0.83	0.87

LPMFCC	Sensitivity	0.58	0.6	0.67
	Specificity	0.64	0.67	0.72
	Precision	0.62	0.64	0.71
	Accuracy	0.61	0.63	0.69
	F1-score	0.6	0.62	0.69

LPCC	Sensitivity	0.54	0.56	0.56
	Specificity	0.6	0.6	0.62
	Precision	0.58	0.58	0.6
	Accuracy	0.57	0.58	0.59
	F1-score	0.56	0.57	0.58

**Table 6:** Comparison of the OSAHS degree of the test result and the OSAHS degree data output in PSG.

Subject number	AHI (PSG)	AHI (test)	SQRT-AHI	Degree (PSG)	Degree (test)
01	5	2	0.75	0	0
02	4.7	0.37	1.08	0	0
03	1.7	6	1.07	0	1
04	2.8	1.7	0.28	0	0
05	1.5	1.7	0.05	0	0
06	41.9	50.3	2.1	3	3
07	25.3	28.1	0.7	2	2
08	7.2	8	0.2	1	1
09	31.7	31.4	0.075	3	3
10	8.6	41	8.1	1	3

## Data Availability

Data are available upon request to the corresponding author.
